# Adoption of Two-Dimensional Ultrasound Gastrointestinal Filling Contrast on Artificial Intelligence Algorithm in Clinical Diagnosis of Gastric Cancer

**DOI:** 10.1155/2022/7385344

**Published:** 2022-04-30

**Authors:** Da Xu, Rong Liu, Huiping Xu, Zhijian Zhang, Wei Li, Yi Zhang, Wenjun Zhang

**Affiliations:** Department of Ultrasound Medicine, Wenjiang District People's Hospital, Chengdu, 611130 Sichuan, China

## Abstract

This research was aimed to explore the value of gastrointestinal filling contrast-enhanced ultrasound (CEUS) and computed tomography (CT-)-enhanced scanning based on artificial intelligence (AI) algorithm in the evaluation of gastric cancer staging. 102 patients with gastric cancer were selected as the research objects. All of them underwent CEUS of gastrointestinal filling and 64-slice spiral CT before surgery. In addition, an improved mean shift algorithm was proposed based on differential optical flow and deep convolutional neural network (D-CNN), which was applied in image processing. The predicted positive rate (PPR), sensitivity, specificity, and accuracy of gastric cancer in different stages by CEUS and CT were calculated using pathological diagnosis results as the gold standard. 17 patients with T1 stage, 41 patients with T2-T3 stage, and 35 patients with T4 stage were detected by CEUS. 13 patients with T1 stage, 34 patients with T2-T3 stage, and 30 patients with T4 stage were detected by CT enhanced examination. The PPRs of CEUS for T1, T2-T3, and T4 stages of gastric cancer were higher than those of CT enhanced (*P* < 0.05). The PPR of CEUS for N0 staging of gastric cancer was higher than that of CT enhanced (*P* < 0.05), and it for N3 staging of gastric cancer was lower than that of CT enhanced (*P* < 0.05). From the analysis of M staging of gastric cancer, the PPRs of CEUS for M0 and M1 staging of gastric cancer were not statistically different from the PPRs of CT enhanced (*P* > 0.05). The sensitivity (95.6%), specificity (81.82%), and accuracy (94.12%) of CEUS in assessing resectability were significantly higher than those of CT enhancement (89.01%, 63.67%, and 86.27%, respectively), and the differences were statistically significant (*P* < 0.05). In summary, CEUS gastrointestinal filling based on the D-CNN algorithm could better improve the display rate of the tissue lesions around the stomach. It also helped to judge the lesion progress, the depth of infiltration, and lymph node metastasis of the lesion. In addition, it had excellent performance in evaluating the resectability of gastric cancer before surgery and had clinical promotion value.

## 1. Introduction

Gastric carcinoma is a malignant tumor that originates from the epithelium of the gastric mucosa. It ranks first among all kinds of malignant tumors in China. There are obvious regional differences in the incidence of gastric cancer. It is higher in the northwest and eastern coastal areas of in China than that in the south [1, 2]. The prevalence is over 50 years old, and the ratio of male to female incidence is 2 : 1. Due to changes in diet, increased work pressure, and helicobacter pylori infection, gastric cancer tends to be younger [3]. Gastric cancer can occur in any part of the stomach, and more than half of them occur in the antrum of the stomach, the greater curvature, the lesser curvature, and the anterior and posterior walls of the stomach [4, 5]. The vast majority of gastric cancer is adenocarcinoma. There are no obvious symptoms in the early stage or nonspecific symptoms such as upper abdominal discomfort and belching. The symptoms are often similar to the symptoms of chronic gastric diseases such as gastritis and gastric ulcer and are easily overlooked. Therefore, the early diagnosis rate of gastric cancer in China is still low. The prognosis of gastric cancer is related to the pathological stage, location, tissue type, biological behavior, and treatment measures of gastric cancer [6]. The gastric cancer can be pathologically classified into early one (the depth of lesion infiltration is limited to the mucosa and submucosa) and advanced one (the lesion invades the submucosa, also called middle and late gastric cancer). Most patients with early gastric cancer have no specific symptoms, so the detection rate is low. Most of the gastric cancer patients found in the clinic are in the middle and advanced stages. The cure rate is extremely low, and the prognosis is very poor. Even if a huge economic cost and a large amount of human resources are paid, the ideal curative effect cannot be obtained [7–9].

With the development of Internet technology and imaging technology, ultrasound technology is gradually applied in the field of clinical diagnosis. However, in the digestive tract organs such as the gastrointestinal tract, the use of ultrasound has encountered great limitations and doubts. The main reason is that these digestive tract organs are all cavity-type organs. The contents and gases contained in the cavity-type organs will interfere with the use of ultrasound to a considerable extent, which will cause great obstacles to the display of the image formed by ultrasound, especially in terms of clarity [10, 11]. The gastrointestinal ultrasound contrast examination method is also called gastrointestinal filling examination method. It fills the gastrointestinal cavity with a contrast agent. After the gastrointestinal cavity was filled with the contrast agent, the ultrasonic image showed an echo similar to that of the solid tissue, eliminating the interference of gas and mucus in the gastric cavity on the gastrointestinal wall and liver, gallbladder, spleen, and pancreas, and producing a significant contrast effect. It does not produce ultrasound artifacts such as the posterior enhanced effect, reverberation effect, and attenuation phenomenon of gastrointestinal cavity and gastrointestinal wall enhanced, which makes up for the deficiency of using anechoic gastrointestinal contrast agent and improves the resolution of the lesion and detection rate [12]. With the development of science and technology, the integration of multiple disciplines has become a general trend. Computer-aided detection has also entered the medical imaging industry. Artificial intelligence (AI) is a new technical science that studies and develops theories, methods, technologies, and application systems used to simulate, extend, and expand human intelligence. It has also been introduced into clinical medical image processing [13, 14]. Therefore, this study intends to introduce artificial intelligence algorithms to enhance contrast ultrasound images.

Convolutional neural network (CNN) is a feedforward neural network with deep structure including convolutional computation and deep structure in deep learning. It is often used in medical image processing and has good computing performance. The differential optical flow method uses the spatiotemporal differentiation of the grayscale of the image sequence (i.e., the spatiotemporal gradient function) to calculate the optical flow of each pixel on the image and assigns a velocity vector to each pixel in the image. According to the velocity vector characteristics of each pixel point, the image can be dynamically analyzed. 102 patients with gastric cancer were selected as the research objects. All patients underwent gastrointestinal filling CEUS examination based on AI algorithms and 64-slice spiral CT enhanced scanning before surgery. The clinical value of probe AI algorithm combined with gastrointestinal filling CEUS in the diagnosis of gastric cancer was evaluated by comparing the diagnostic results of the two methods on the staging and resectability of gastric cancer.

## 2. Materials and Methods

### 2.1. Research Objects

One hundred and two patients with gastric cancer were selected from hospital from January 2019 to June 2021 as the research objects. There were 73 males and 29 females, aged 26-78 years old. All patients underwent gastrointestinal filling CEUS examination and 64-slice spiral CT scan before surgery. The study had been approved by the medical ethics committee of hospital. The patients and their families knew about the study and signed the informed consent form.

Inclusion criteria are as follows: (1) repeated upper abdominal pain or discomfort with fullness; (2) unexplained weight loss or anemia; (3) intermittent hematemesis or melena; (4) gastric cancer confirmed by gastroscopy; and (5) before admission, any anti-inflammatory and anticancer treatments were not received.

Exclusion criteria are as follows: (1) patients with severe pyloric obstruction; (2) combined intestinal obstruction; (3) patients with pancreatitis; (4) patients with gastrointestinal perforation and gastric dilatation; (5) incomplete clinical data; and (6) withdrawing midway experimental patient.

### 2.2. Gastrointestinal Filling CEUS

Color Doppler ultrasound was used. The probe is a conventional abdominal probe, and the frequency is 3.5-5.5 MHZ. The fast-dissolving gastrointestinal ultrasound aid was applied. About 450 mL of 95°C boiled water and 45 g of contrast medium were mixed and put into the container. A uniform thin paste liquid was formed after stirring. After it was cooled to the appropriate temperature and given orally to the patient, ultrasonic examination could be carried out. If necessary, ultrasonic examination could be carried out while taking it.

The patients were required to fast for 8 hours and to have no water for 4 hours. The patients were asked to have a light diet for dinner the day before, and not eat gas-producing food. Fasting routine examination was performed. The patient was instructed to lie flat. The gall bladder, spleen, pancreas, kidney, abdominal cavity, retroperitoneum, and gastrointestinal areas were scanned with probes. From the lower esophagus, cardia, gastric fundus, gastric body curvature, anterior and posterior wall, gastric angle, and gastric antrum to duodenum were scanned.

### 2.3. Enhanced Spiral CT Scan

128-slice spiral CT was used. The contrast agent was used, the amount of contrast agent was calculated at 1.5 mL/kg, and the intravenous injection rate was 2.5-3 mL/s. The patient was asked to take a supine position. CT scan was performed from the top of the diaphragm to the lower contour of the stomach. In addition, the enhanced two-phase scan was performed.

### 2.4. Target Tracking Algorithm Based on Differential Optical Flow and CNN

Particle filter was based on Monte Carlo method [15], and the idea of resampling was added. A set of samples (particles) was used to approximate the posterior probability distribution of the system, and then, this approximate representation was used to estimate the state of the nonlinear system. However, in the resampling stage, the diversity and effectiveness of particles were prone to be low. Therefore, how to improve the resampling method, increase the diversity of particles, and increase the calculation of weights were particularly important.

In this work, a target tracking algorithm based on differential optical flow and convolution neural network is proposed. Firstly, the particle trajectory is evaluated by optical flow method [16]. Then, the edge information of particles was extracted by deep convolution neural network [17]. Finally, the final position was judged by classification. The basic flow of the algorithm is shown in Figure 1 below.

Before the focus target was tracked, the target rectangle needed to be manually selected as the area to be tracked in the original image. Then, multiscale Retinex with chromaticity preservation (MSRCP) algorithm [18] was used to preprocess the image to obtain the enhanced image. Hue-saturation-value (HSV) color space model was used to extract image features. The image was converted from red-green-blue (RGB) space to HSV space. The conversion equation of each color could be *H*_colour_ = *I*_colour_(*RGB*_colour_). Then, the transformation equation of *H*, *S*, and *V* spaces could be expressed as follows:

(1) $$\begin{array}{c} V=\max\left(R,G,B\right),\\ S⟵\frac{\left(\max\left(R,G,B\right)-\min\left(R,G,B\right)\right)}{\max\left(R,G,B\right)}. \end{array}$$

The conversion of H space had to be carried out according to conditions: when *V* = *R*, *H*⟵60∗(*G*‐*B*)/(max(*R*, *G*, *B*) − min(*R*, *G*, *B*)); when *V* = *G*, *H*⟵(120 + 60∗(*G*‐*B*))/(max(*R*, *G*, *B*) − min(*R*, *G*, *B*)); and when *V* = *B*, *H*⟵(240 + 60∗(*G*‐*B*))/(max(()) − min(*R*, *G*, *B*)).

Random particles were put in the target area to be tracked. The optical flow component of each particle area was calculated. The weight value of each particle was obtained. According to the weight, the particle position was divided to determine multiple candidate areas (Figure 2).

The optical flow component of the current frame was generally not obtained during the calculation. Thus, multiple particles were randomly selected in the previous frame, the optical flow component of each particle was calculated, and the optical flow field of the current frame was obtained. It was assumed that the characteristic point of the last frame of image was (*m*_*i*_, *n*_*j*_), the speed of the image at this point was the optical flow of the pixel, and the optical flow components could be superimposed to obtain

(2) $$\begin{array}{c} \text{sum }\left(m\right)=\underset{i}{\sum }\underset{j}{\sum }\frac{di}{dt}, \end{array}$$

(3) $$\begin{array}{c} \text{sum }\left(n\right)=\underset{i}{\sum }\underset{j}{\sum }\frac{dj}{dt}. \end{array}$$

Equations (2) and (3) are changed again to get

(4) $$\begin{array}{c} h_{s}={\left[\text{sum}\left(m\right),\text{sum}\left(n\right)\right]}^{T}, \end{array}$$

(5) $$\begin{array}{c} w_{s}=\sqrt{\frac{\text{sum}{\left(m\right)}^{2}+\text{sum}{\left(n\right)}^{2}}{z}}, \end{array}$$

where *z* represents the pixel, *s* represents the *s*-th frame of the image, *h* represents the total optical flow, and *w* represents the optical flow motion intensity of the image. From the above calculation, the optical flow component of the *s*-th frame could be obtained, and the component equations could be changed to obtain

(6) $$\begin{array}{c} h_{\alpha }=h_{s-1}\left(1-\beta \right)+\beta h_{s}, \end{array}$$

(7) $$\begin{array}{c} w_{\alpha }=w_{s}, \end{array}$$

where *β* represents the update factor and *h*_*α*_ and *w*_*α*_ represent the optical flow model after the current frame was updated. It was assumed that each particle region was *R*_*k*_ = [*sum*(*m*_*k*_), *sum*(*n*_*k*_)]^*T*^. The similarity between the particle region and the target region was evaluated. Equation (8) could be obtained. The particle weight value of the current frame is calculated by using Equation (8), and Equation (9) could be obtained.

(8) $$\begin{array}{c} \text{Consi}\left({R_{\alpha }}^{\prime },R_{k}\right)=\frac{{R_{k}}^{T}*{R_{\alpha }}^{\prime }*\left|R_{k}\right|}{{R_{\alpha }}^{\prime }}, \end{array}$$

(9) $$\begin{array}{c} q^{i}=\frac{\exp\langle -\text{Consi}\left({R_{\alpha }}^{\prime },R_{k}\right)-{\left(\text{Consi}\left({R_{\alpha }}^{\prime },R_{k}\right)\right)}^{2}/2{\pi \varepsilon }^{2}\rangle }{\sqrt{2\pi \varepsilon }}, \end{array}$$

where *ε*^2^ represents the squared difference, *q*^*i*^ represents the particle weight value, and Consi(*R*_*α*_′, *R*_*k*_) represents the similarity between the particle area and the target area.

The particles were updated, and more particles were placed in places with large weights. Fewer particles were placed in other areas. The target candidate area *Q* was determined according to the position of the particle, namely, [*Q*_1_, *Q*_2_, ⋯, *Q*_*n*_]. Finally, the CNN was introduced to process the candidate samples, and the size of the candidate particle area was normalized to the same size by means of scale normalization. The generated candidate target rectangular box was input into CNN, and the features were output after feature extraction vector. The representative feature vectors such as edge contours extracted in the previous step were used as the input of the discriminant classifier, and finally, the classification result was obtained. The target tracking algorithm based on differential optical flow and CNN in this article was set as D-CNN.

### 2.5. Simulation Experiment

The experimental simulation platform is as follows: The operating system is Window10, the memory size is 12GB, the CPU is I5 7500 (3.4Hz), the graphics card is Tesla K40c, and the software is Matlab9.1 (MathWorks, USA).

CNN model was introduced. MSRCP algorithm and D-CNN algorithm were compared. The average center location error (CLE), target overlap area ratio (TOAR), and similarity (SI) were used as evaluation indicators [19].

1. CLE referred to the center coordinates of the rectangular frame of the tracking result of each frame of image in the tracking process. The pixel distance from the center point of the real lesion area was calculated. The center errors of all marked pictures in a video were summed. The average value of the video sequence error was calculated. The greater the distance was, the greater the error was
2. The equation of TOAR could be expressed as follows

ROD represented the relative degree of overlap between the segmentation result and the actual target, which could be expressed as follows:

(10) $$\begin{array}{c} \text{TOAR}=.\left|\frac{\text{area}\left(s_{a}\cap s_{b}\right)}{\text{area}\left(s_{a}\cup s_{b}\right)}\right|. \end{array}$$

The SI equation could be expressed as follows:

(11) $$\begin{array}{c} SI=\sqrt{1-\underset{P}{\sum }\frac{H_{1}\left(P\right)H_{2}\left(P\right)}{\sum_{P}H_{1}\left(P\right)\sum_{P}H_{2}\left(P\right)}}, \end{array}$$

where *s*_*a*_ represents the area of the real tracking area, *s*_*b*_ represents the area of the tracking area obtained by the algorithm, *H*_1_ represents the first frame of the contrast image, *H*_2_ represents the 2-nth frame of the contrast image, and *P* represents the probability distribution of image pixel gray values.

### 2.6. Statistical Methods

The data processing of this study was analyzed by SPSS19.0 version statistical software, the measurement data was expressed by the mean ± standard deviation (−*x* ± *s*), and the count data was expressed by the percentage (%). One-way analysis of variance was used for pairwise comparison. The difference was statistically significant at *P* < 0.05.

## 3. Results

### 3.1. Analysis of Experimental Results

Figure 3 illustrates that the difference between D-CNN algorithm and other algorithms in average center error, target overlap area ratio, and similarity index was statistically significant. The average center error and similarity index of D-CNN algorithm were significantly less than CNN and MSRCP algorithm, and the target overlap area ratio is obviously greater than CNN and MSRCP algorithm (*P* < 0.05).

Figures 4 and 5 are the 15th and 102th frames of the CEUS images. The green dots represented the tracked motion trajectory, and the blue rectangle represented the position predicted by the algorithm. The target tracking results of the whole image from different algorithms showed that the tracking position predicted by D-CNN algorithm was the closest to that marked by experts, while there was a certain deviation between the predicted position of MSRCP algorithm and CNN algorithm and that marked by experts.

### 3.2. Patient Clinical Data

Figure 6 indicates that 21 cases of gastric corpus, 36 cases of gastric antrum, 18 cases of gastric horn, 22 cases of cardia, and 5 cases of gastric fundus were included in the patient's lesions. 26 cases of early gastric cancer and 76 cases of advanced gastric cancer were included.

A 56-year-old male, diagnosed with gastric cancer by gastroscope, refused the gastroscope review after coming to the hospital and performed CEUS examination. Ultrasound images showed that the stomach was well filled. The gastric wall on the side of the cardia gastric curvature was diffusely thickened and appeared hypoechoic, with local masses and nodules, and no obvious boundary with the normal gastric wall was found. The normal hierarchical structure of the local gastric wall disappeared, and the masses grew outward. There was no obvious adhesion with surrounding organs (Figure 7).

A 68-year-old woman came to see the doctor with an upset stomach for one month. Ultrasound images showed in Figure 8 that the mucosa of the gastric wall at the corner of the lesser curvature of the stomach is locally bulging, with reduced echo, disordered levels, with a range of 2.83 cm, and a thickening of about 1.49 cm. There were multiple enlarged lymph nodes in the abdominal cavity around the stomach.

### 3.3. Diagnosis Results of T Staging of Gastric Cancer

The pathological results showed in Figure 9(a) that there are 19 patients with T1 stage, 45 patients with T2-T3 stage, and 38 patients with T4 stage. The CEUS showed that there were 17 patients with T1 stage, 41 patients with T2-T3 stage, and 35 patients with T4 stage. CT-enhanced examination showed that there were 13 patients with T1 stage, 34 patients with T2-T3 stage, and 30 patients with T4 stage.

Further comparison of the positive rate (Figure 9(b)) showed that the positive rates of CEUS for T1, T2-T3, and T4 stages of gastric cancer were all higher than those of CT enhanced, and the difference was statistically significant (*P* < 0.05).

### 3.4. Diagnosis Results of N Staging of Gastric Cancer

The pathological results (Figure 10(a)) showed that there were 42 patients with N0 stage, 16 patients with N1 stage, 21 patients with N2 stage, and 23 patients with N3 stage. CEUS revealed there were 39 patients with N0 stage, 11 patients in stage N1, 15 patients in N2 stage, and 11 patients in N3 stage; CT enhanced examination showed that there were 31 patients in N0 stage, 12 patients in N1 stage, 16 patients in N2 stage, and 17 patients in N3 stage.

Further comparison of the positive rate (Figure 10(b)) showed that the predicted positive rate (PPR) of CEUS for N0 staging of gastric cancer was higher than that of CT enhanced and the difference was statistically significant (*P* < 0.05). The PPR of CEUS for N3 staging of gastric cancer was lower than CT enhanced, and the difference was statistically significant (*P* < 0.05). Compared with CT enhanced, the positive rate of CEUS in N1 and N2 staging of gastric cancer was not statistically significant (*P* > 0.05).

### 3.5. Diagnosis Results of M Staging of Gastric Cancer

The pathological results (Figure 11(a)) showed that there were 68 patients with M0 stage and 34 patients with M1 stage. There were 68 patients with M0 stage and 31 patients with M1 stage detected by CEUS. CT-enhanced examination showed that there were 68 patients with M0 stage and 29 patients with M1 stage.

Further comparison of the PPR of examination (Figure 10(b)) showed that the PPR of CEUS for M0 and M1 staging of gastric cancer was not statistically different from CT enhanced (*P* > 0.05).

### 3.6. Evaluation of Resectability by CEUS and Computed Tomography

In the postoperative pathological results (Figures 12(a) and 12(b)), there were 91 resectable patients and 11 unresectable patients. Among the 91 resectable patients, the CEUS judgment was accurate in 87 cases, and the misjudgment was 4 cases. The CT-enhanced judgment was accurate in 81 cases, and the misjudgment was 10 cases. Among the 11 unresectable patients, the CEUS judgment was accurate in 9 cases, and the misjudgment was 2 cases. The CT enhanced judgment was accurate in 7 cases, and the misjudgment was 4 cases.

Figure 12(c) shows that the sensitivity, specificity, and accuracy of CEUS in assessing resectability were significantly higher than those of CT enhanced and the difference was statistically significant (*P* < 0.05).

## 4. Discussion

Gastric cancer belongs to the category of genetic disease. The oncogenes and anticancer genes involve in the occurrence and development of gastric cancer. Under the action of many factors, normal gastric mucosal tissue is subjected to a variety of cancer-promoting effects in various stages, resulting in excessive proliferation of gastric epithelial cells and finally transformed into cancer tissue. With the rapid development of computer technology at present, the clinical diagnosis of gastric cancer tends to be more intelligent and accurate. Although ultrasound is a commonly used means in clinic, it has poor effect in gastrointestinal organs such as gastrointestinal tract. This situation did not end until the gastrointestinal ultrasound contrast agent and ultrasonic gastrointestinal filling angiography were put into use [20–22]. At present, it is still a hot topic to study the application effect of gastrointestinal filling CEUS and CT enhanced scanning in the staging evaluation of gastric cancer. In this study, 102 patients with gastric cancer were selected as the research objects, and gastrointestinal filling CEUS and 64-slice spiral CT enhanced scanning were performed before operation. Moreover, based on differential optical flow and convolution neural network, a focus target tracking algorithm D-CNN algorithm was proposed for image enhanced. Firstly, CNN algorithm and MSRCP algorithm were introduced and compared with the algorithm proposed in this study. It was found that the average center error, target overlap area ratio, and similarity index of D-CNN algorithm were statistically significant compared with other algorithms. The index data were better than CNN and MSRCP algorithm (*P* < 0.05). This showed from the quantitative data that the focus target tracking performance of D-CNN algorithm in ultrasonic image was better than that of traditional algorithm to a certain extent, and the error rate and overlapping area rate were the lowest. In addition, it was found that from the adoption on the actual CEUS images that the tracking position predicted by D-CNN algorithm was the closest to that marked by experts, while there was a certain deviation between the predicted position of msrcp algorithm and CNN algorithm and that marked by experts. Contrast-enhanced ultrasonography based on D-CNN algorithm was applied to the staging evaluation of gastric cancer patients.

It was found that 17 patients with T1 stage, 41 patients with T2-T3 stage, and 35 patients with T4 stage were examined by contrast-enhanced ultrasonography. 13 patients with T1 stage, 34 patients with T2-T3 stage, and 30 patients with T4 stage were detected by CT enhanced. This was different from the study of Liu JJ (2020) et al. [23]. The reason may be that 3 of the missed cases belonged to the category of micro gastric cancer, the gastric wall had no obvious thickening, and no micro lesions were scanned by CEUS and enhanced CT. The pathological was taken as the gold standard. It was found that the positive rate of contrast-enhanced ultrasonography in T1, T2-T3, and T4 staging of gastric cancer was higher than that of enhanced CT, and the difference was statistically significant (*P* < 0.05), which showed that the diagnostic performance of gastrointestinal filling angiography in T staging of gastric cancer was better than that of enhanced CT. As for the cases with inaccurate diagnosis in CEUS, there are three possible reasons. First, the probe sound beam was not perpendicular to the gastric wall due to the inflammatory reaction of the tissue around the cancerous site, the level of gastric wall was blurred, and the judgment stage was too high. Second, it is difficult to distinguish the small tumor and hyperechoic serosa of gastric wall from its adjacent tissues, which makes the judgment of staging too low. Third, canceration is often accompanied by ulcer. When fibrosis occurs at the bottom of the ulcer, the hierarchical structure of the gastric wall disappears, and the judgment stage is too high [24].

From the analysis of N staging, the positive rate of CEUS in N0 staging of gastric cancer was higher than that of CT enhanced, and the difference was statistically significant (*P* < 0.05). It showed that contrast-enhanced ultrasonography of gastrointestinal filling had a high diagnostic value in N0 staging of gastric cancer. However, the positive rate of contrast-enhanced ultrasonography in N3 staging of gastric cancer was lower than that of CT enhanced, and the difference was statistically significant (*P* < 0.05). Such result is different from the argument made by Joo I (2019) et al. [25], who explored the correlation between contrast agent-enhanced ultrasound parameters and perfusion CT (PCT) parameters in gastric cancer, which may be caused by more metastatic lymph nodes in gastric body and fundus or multiple inflammatory lymph nodes in the included patients. It is not conducive to the examination of gastrointestinal filling CEUS [26]. The analysis of M-stage of gastric cancer revealed that there was no significant difference in the positive rate of contrast-enhanced ultrasonography in M0 and M1 stages of gastric cancer compared with enhanced CT (*P* > 0.05). It showed that the value of gastrointestinal filling CEUS and enhanced CT in the evaluation of M-stage of gastric cancer was the same, and there was no significant difference. It was found that the sensitivity, specificity, and accuracy of gastrointestinal filling CEUS in evaluating the resectability of gastric cancer were significantly higher than those of CT enhanced, and the difference was statistically significant (*P* < 0.05). It indicates that gastrointestinal filling CEUS has high sensitivity and specificity in evaluating the resectability of gastric cancer before operation. It can objectively be used as one of the main auxiliary examinations for the preoperative evaluation of resectability of gastric cancer.

## 5. Conclusion

In this work, 102 patients with gastric cancer were selected as the research object. Before operation, gastrointestinal filling CEUS and 64-slice spiral CT were performed. In addition, a lesion target tracking algorithm D-CNN algorithm was proposed based on differential optical flow and convolutional neural network for image enhanced. It was found that gastrointestinal filling CEUS based on D-CNN algorithm could better improve the display rate of lesions around the stomach and help to judge the lesion process, depth of invasion, and lymph node metastasis. Moreover, it also had excellent performance in the preoperative resectability evaluation of gastric cancer, which was of clinical value. However, there are few patients included in this work, so more samples need to be accumulated in the back for in-depth probe. In addition, there is no unified standard for the patient's body position, body shape, and section angle during imaging examination. Later, it will increase the inclusion of research samples and further explore the application of imaging and AI algorithms in clinical screening of gastric cancer. It is necessary to improve it in the follow-up. In conclusion, the research content of this study provides a data reference for the clinical application of gastrointestinal filling CEUS at a certain level.

## Figures and Tables

**Figure 1:** Flow chart of target tracking algorithm based on differential optical flow and CNN.

**Figure 2:** The calculation process of particle weight heavy stock value.

**Figure 3:** Comparison of tracking performance indicators of different algorithms for CEUS images. # indicated that the difference compared with the D-CNN algorithm was statistically significant (*P* < 0.05).

**Figure 4:** Algorithmic prediction results of the 15th frame of CEUS image. (a) The expert annotation; (b) the D-CNN algorithm; (c) the MSRCP algorithm; and (d) the CNN algorithm.

**Figure 5:** Algorithmic prediction results of the 102nd frame of CEUS image. (a) The expert annotation; (b) the D-CNN algorithm; (c) the MSRCP algorithm; and (d) the CNN algorithm.

**Figure 6:** Clinical data of the patient. (a) The lesion site. (b) The pathological type.

**Figure 7:** Different sections of CEUS images of a gastric cancer patient (male, 52 years old).

**Figure 8:** Different sections of CEUS images of a gastric cancer patient (female, 68 years old).

**Figure 9:** Diagnosis results of T staging of gastric cancer. (a) The number of T1, T2-3, and T4 staging examinations. (b) The positive rate of examinations. ∗ indicated that the difference was statistically significant compared with CEUS (*P* < 0.05).

**Figure 10:** Diagnosis results of N staging of gastric cancer. (a) The number of N0, N1, N2, and N3 staging examinations. (b) The PPR of examinations. ∗ indicated that the difference was statistically significant compared with CEUS (*P* < 0.05).

**Figure 11:** Diagnosis results of M staging of gastric cancer. (a) The number of cases examined by M0 and M1 staging. (b) The PPR of examination.

**Figure 12:** CEUS and CT enhanced for the assessment of resectability. (a) The assessment of resectable patients; (b) the assessment of unresectable patients; and (c) the assessment of sensitivity, specificity, and accuracy. ∗ meant the difference was statistically significant compared with CEUS (*P* < 0.05).

## Data Availability

The data used to support the findings of this study are available from the corresponding author upon request.

## References

[1] Machlowska J., Baj J., Sitarz M., Maciejewski R., Sitarz R. (2020). Gastric cancer: epidemiology, risk factors, classification, genomic characteristics and treatment strategies. *International Journal of Molecular Sciences*.

[2] Tan Z. (2019). Recent advances in the surgical treatment of advanced gastric cancer: a review. *Medical Science Monitor*.

[3] Engstrand L., Graham D. Y. (2020). Microbiome and gastric cancer. *Digestive Diseases and Sciences*.

[4] Li Y., Zhao J. L., Lv Z. H., Li J. H. (2021). Medical image fusion method by deep learning. *International Journal of Cognitive Computing in Engineering.*.

[5] Ford A. C., Yuan Y., Moayyedi P. (2020). Helicobacter pylorieradication therapy to prevent gastric cancer: systematic review and meta-analysis. *Gut*.

[6] Tsukamoto T., Nakagawa M., Kiriyama Y., Toyoda T., Cao X. (2017). Prevention of gastric cancer: eradication of helicobacter pylori and beyond. *International Journal of Molecular Sciences*.

[7] Uno Y. (2019). Prevention of gastric cancer by Helicobacter pylori eradication: a review from Japan. *Cancer Medicine*.

[8] Shao L., Li P., Ye J. (2018). Risk of gastric cancer among patients with gastric intestinal metaplasia. *International Journal of Cancer*.

[9] Herzberg M., Beer M., Anupindi S., Vollert K., Kröncke T. (2018). Imaging pediatric gastrointestinal stromal tumor (GIST). *Journal of Pediatric Surgery*.

[10] Lv Z., Qiao L., Wang Q., Piccialli F. (2021). Advanced machine-learning methods for brain-computer interfacing. *IEEE/ACM Transactions on Computational Biology and Bioinformatics*.

[11] Jiang Y., Wang H., Wu J. (2020). Noninvasive imaging evaluation of tumor immune microenvironment to predict outcomes in gastric cancer. *Annals of Oncology*.

[12] He P., Miao L. Y., Ge H. Y. (2019). Preoperative tumor staging of gastric cancer: comparison of double contrast-enhanced ultrasound and multidetector computed tomography. *Journal of Ultrasound in Medicine*.

[13] Hu M., Zhong Y., Xie S., Lv H., Lv Z. (2021). Fuzzy system based medical image processing for brain disease prediction. *Frontiers in Neuroscience*.

[14] Renzulli M., Clemente A., Spinelli D. (2020). Gastric cancer staging: is it time for magnetic resonance imaging?. *Cancers*.

[15] Huang Z., Liu D., Chen X. (2020). Retrospective imaging studies of gastric cancer: study protocol clinical trial (SPIRIT Compliant). *Medicine*.

[16] Sun Z. Q., Hu S. D., Li J., Wang T., Duan S. F., Wang J. (2019). Radiomics study for differentiating gastric cancer from gastric stromal tumor based on contrast-enhanced CT images. *Journal of X-Ray Science and Technology*.

[17] Yan C. X., Huang P. T., Shentu W. H. (2018). Value of double contrast-enhanced ultrasound QontraXt three-dimensional pseudocolor quantitative analysis to therapeutic effect evaluation of preoperative neoadjuvant chemotherapy in advanced gastric cancer patients. *Zhonghua Zhong Liu Za Zhi*.

[18] Tang L., Wang X. J., Baba H., Giganti F. (2020). Gastric cancer and image-derived quantitative parameters: part 2-a critical review of DCE-MRI and 18F-FDG PET/CT findings. *European Radiology*.

[19] Giganti F., Tang L., Baba H. (2019). Gastric cancer and imaging biomarkers: part 1- a critical review of DW-MRI and CE-MDCT findings. *European Radiology*.

[20] Wang X., Kou H., He H., Lu M., Zhou L., Wang L. (2020). Difference in perfusion parameters between gastric cancer and gastric stromal tumors: evaluation with oral contrast plus contrast-enhanced ultrasonography. *Frontiers in Oncology*.

[21] Wang L., Liu Z., Kou H. (2019). Double contrast-enhanced ultrasonography in preoperative T staging of gastric cancer: a comparison with endoscopic ultrasonography. *Frontiers in Oncology*.

[22] Tsurumaru D., Nishimuta Y., Muraki T. (2019). CT gastrography “wall-carving technique” of gastric cancer: impact of contrast enhancement based on layer depth. *Japanese Journal of Radiology*.

[23] Liu J. J., Liu W., Jin Z. Y. (2020). Improved visualization of gastric cancer and increased diagnostic performance in lesion depiction and depth identification using monoenergetic reconstructions from a novel dual-layer spectral detector CT. *Academic Radiology*.

[24] Ji L., Liu Z., Zhou B. (2020). Community-based pilot study of a screening program for gastric cancer in a Chinese population. *Cancer Prevention Research (Philadelphia, Pa.)*.

[25] Schellhaas B., Bernatik T., Bohle W. (2021). Contrast-enhanced ultrasound algorithms (CEUS-LIRADS/ESCULAP) for the noninvasive diagnosis of hepatocellular carcinoma – a prospective multicenter DEGUM study. *Ultraschall in der Medizin*.

[26] Zamani M., Skagen K., Scott H., Lindberg B., Russell D., Skjelland M. (2019). Carotid plaque neovascularization detected with superb microvascular imaging ultrasound without using contrast media. *Stroke*.

